# Acetylshikonin Sensitizes Hepatocellular Carcinoma Cells to Apoptosis through ROS-Mediated Caspase Activation

This article has been retracted.

**DOI:** 10.3390/cells8111466

**Published:** 2019-11-19

**Authors:** Ming Hong, Jinke Li, Siying Li, Mohammed M.Almutairi

**Affiliations:** 1 Science and Technology Innovation Center, Guangzhou University of Chinese Medicine, Guangzhou 51000, China; 2 Institute of Clinical Pharmacology, Guangzhou University of Chinese Medicine, Guangzhou 51000, China; 3 Department of Pharmacology & Toxicology, University of Kansas, Lawrence, KS 66045, USA; j086l791@ku.edu (J.L.); s070l205@ku.edu (S.L.)

**Keywords:** acetylshikonin, apoptosis-resistant, hepatocellular carcinoma, caspase activation

## Abstract

The tumor necrosis factor-related apoptosis-inducing ligand (TRAIL) has shown strong and explicit cancer cell-selectivity, which results in little toxicity toward normal tissues, and has been recognized as a potential, relatively safe anticancer agent. However, several cancers are resistant to the apoptosis induced by TRAIL. A recent study found that shikonin b (alkannin, 5,8-dihydroxy-2-[(1*S*)-1-hydroxy-4-methylpent-3-en-1-yl]naphthalene-1,4-dione) might induce apoptosis in TRAIL-resistant cholangiocarcinoma cells through reactive oxygen species (ROS)-mediated caspases activation. However, the strong cytotoxic activity has limited its potential as an anticancer drug. Thus, the current study intends to discover novel shikonin derivatives which can sensitize the liver cancer cell to TRAIL-induced apoptosis while exhibiting little toxicity toward the normal hepatic cell. The trypan blue exclusion assay, western blot assay, 4′,6-diamidino-2-phenylindole (DAPI) staining and the terminal deoxynucleotidyl transferase dUTP nick end labeling (TUNEL) assay as well as the ‘comet’ assay, were used to study the underlying mechanisms of cell death and to search for any mechanisms of an enhancement of TRAIL-mediated apoptosis in the presence of ASH. Herein, we demonstrated that non-cytotoxic doses of acetylshikonin (ASH), one of the shikonin derivatives, in combination with TRAIL, could promote apoptosis in HepG2 cells. Further studies showed that application of ASH in a non-cytotoxic dose (2.5 μM) could increase intracellular ROS production and induce DNA damage, which might trigger a cell intrinsic apoptosis pathway in the TRAIL-resistant HepG2 cell. Combination treatment with a non-cytotoxic dose of ASH and TRAIL activated caspase and increased the cleavage of PARP-1 in the HepG2 cell. However, when intracellular ROS production was suppressed by N-acetyl-l-cysteine (NAC), the synergistic effects of ASH and TRAIL on hepatocellular carcinoma (HCC) cell apoptosis was abolished. Furthermore, NAC could alleviate p53 and the p53 upregulated modulator of apoptosis (PUMA) expression induced by TRAIL and ASH. Small (or short) interfering RNA (siRNA) targeting PUMA or p53 significantly reversed ASH-mediated sensitization to TRAIL-induced apoptosis. In addition, Bax gene deficiency also abolished ASH-induced TRAIL sensitization. An orthotopical HCC implantation mice model further confirmed that co-treated ASH overcomes TRAIL resistance in HCC cells without exhibiting potent toxicity in vivo. In conclusion, the above data suggested that ROS could induce DNA damage and activating p53/PUMA/Bax signaling, and thus, this resulted in the permeabilization of mitochondrial outer membrane and activating caspases as well as sensitizing the HCC cell to apoptosis induced by TRAIL and ASH treatment.

## 1. Introduction

Hepatocellular carcinoma (HCC) is one of the most common human malignancies worldwide, especially in Asian courtiers. Despite the remarkable progress in HCC management, it is still one of the most highly aggressive tumors, with dismal prognosis due to recurrence and metastasis [1,2]. In recent decades, several candidate drugs have been promisingly developed for the patients who cannot be cured by surgical resection. However, it is still necessary to find more potent chemotherapeutics with less side effects and reduced drug resistance in the future medical management of HCC. On that case, several novel molecular target agents have been developed for specifically interfering with HCC growth and metastases while sparing normal cells, such as the tumor necrosis factor-related apoptosis-inducing ligand (TRAIL) [3,4]. TRAIL can trigger the apoptosis cascades by activating death receptors in the cell membrane and inducing the activation of initiator caspase in the extrinsic apoptosis pathway [5]. Although TRAIL is a promising antitumor agent, various cancer cell lines, including HCC cell lines, develop resistance to TRAIL-induced apoptosis [6,7]. Thus, researchers are trying to discovery novel drugs to sensitize the HCC cell to TRAIL-induced apoptosis, while sparing normal cells and tissues.

Shikonin is a natural active ingredient isolated form *Lithospermum erythrorhizon*. Previous studies showed that shikonin and its derivatives could significantly inhibit oxidative stress and attenuated hepatic inflammatory response, as well as protect chronic liver injury [4,5]. Chronic hepatic damage may promote the initiation and development of liver cancer, therefore, the potential hepatoprotective effects of shikonin and its derivatives in hepatitis indicate that these agents may also exert prevention or therapeutic effects in HCC. In recent decades many researches have demonstrated that shikonin might exhibit anti-cancer potential in various kinds of cancer, such as breast cancer, lung cancer, acute myeloid leukemia and HCC [4,8,9]. Interestingly, a recent study found that shikonin (10 µM) might reduce cells’ survival rate and promote apoptosis in cholangiocarcinoma cells, and the suppressive effects could be enhanced by TRAIL treatment through reactive oxygen species (ROS)-mediated caspases activation [7]. However, as a reversible inhibitor of the Uridine 5’-diphospho-glucuronosyltransferase enzyme, shikonin has a high risk of inducing hepatic and renal toxicity [10]. Thus, the strong cytotoxic activity and possible side effects have limited its potential as an anticancer drug [11,12,13]. Recently, several shikonin derivatives with relatively few side effects and minimal toxicity have been developed as potential chemotherapeutic agents against human cancer, such as acetylshikonin (ASH) [14]. ASH is less cytotoxic than shikonin to normal cells, and it can be concluded that ASH may be a potentially safer alternative to shikonin for cancer treatment [14,15]. Previous studies have shown that 10 μM ASH could induce ROS production and enhance the phosphorylation of p38 mitogen-activated protein kinase (MAPK) and c-Jun N-terminal kinase (JNK), which are in the major pathways of apoptotic cell death [15]. Another study has demonstrated that 10 μM ASH could sensitize HCC cells to apoptosis by activating p53, Bax, and Caspase3 [16]. In addition, ASH (10 μM) inhibited the growth of human gastric carcinoma SGC-7901 cells in vitro and in vivo by inducing PUMA-dependent cell apoptosis, which indicated that ASH might sensitize tumor cells to apoptosis [17]. Although ASH has been found to be less toxic than shikonin, 10 μM ASH still has potential cytotoxicity towards normal cells [14]. Thus, we intend to treat HCC with relatively low doses of ASH in combination with TRAIL for evaluating the potential sensitizing effect of ASH to TRAIL-induced apoptosis.

Reactive oxygen species (ROS) can promote cells apoptosis via inducing DNA damage and subsequently activating down-stream signal pathways. For instance, ROS can activate p53 and induce apoptosis via the p53 up-regulated modulator of apoptosis (PUMA) up-regulation, as well as promoting Bax translocation to mitochondria [2,18]. As a BH3-only pro-apoptotic Bcl-2 family protein, PUMA can induce apoptotic cell death by translocation to mitochondria and promote various pro-apoptotic members’ activation, such as Bax. Bax will facilitate Cytochrome C release from mitochondria and activate Caspase. ROS production and DNA damage can directly activate p53 and promote PUMA transcription, which finally induces cell apoptosis [19].

Previous research has shown that ASH (10 μM) could suppress tumor development by inducing PUMA-dependent cell apoptosis [17]. P53/PUMA/Bax activation may be involved in the cell-intrinsic apoptosis pathway by ASH and exhibit synergistic effects with TRAIL-induced cell-extrinsic apoptosis in HCC cells.

In an effort to identify the synergistic effect of ASH and TRAIL in HCC cell apoptosis, we examined whether ASH (non-cytotoxic dosage) in combination with TRAIL could induce apoptotic cell death in a HepG2 cell. Our results demonstrated that ASH (2.5 μM) could reverse the TRAIL resistance in the HepG2 cell. ROS production, DNA double-strand breaks and p53-induced PUMA and Bax activation may contribute to the sensitization effects of ASH on TRAIL-induced apoptosis. We considered that both cellular intrinsic (p53/PUMA/Bax) and extrinsic (TRAIL) pathways contributed to HepG2 cells’ apoptosis via the synergistic antitumor effects of ASH and TRAIL.

## 2. Methods

### 2.1. Reagents and Cell Culture

Human hepatocellular carcinoma cells HepG2, Huh7 and normal hepatic cell LO2 were provided by Dr. Wu in The University of Kansas. Wild-type and p53−/−Hep3B cells, wild-type and p53 upregulated modulator of apoptosis (PUMA)−/−Hep3B cells, HepG2 Bax+/− and HepG2 Bax−/− Cells were provided by Prof. Shi in the University of Kansas. Cells were grown in Roswell Park Memorial Institute (RPMI) 1640 supplemented with penicillin (5 units/mL), streptomycin (5 ug/mL), and 10% heat-inactivated fetal bovine serum (FBS). Acetylshikonin was obtained from Huakang Pharmaceutical Company (Deyang, China) and resolved in 0.1% dimethyl sulfoxide (DMSO). zlETD-fmk, zlEHD-fmk, zDEVD-fmk and N-acetyl-l-cysteine (NAC) were purchased from Sigma-Aldrich Corp (St. Louis, MO, USA). Recombinant human tumor necrosis factor-related apoptosis-inducing ligand (TRAIL) was purchased from R&D Systems (Wiesbaden, Germany) and resolved in PBS + 0.01% bovine serum albumin (BSA).

### 2.2. Cell Viability

Hepatocellular carcinoma (HCC) cells were cultured in a 6-well microplate for 48 h, where each well contain 1 × 10^4^ cells. For the Trypan blue exclusion assay, cells were trypsinized and re-suspended in 0.3 mL DMEM medium, 0.5 mL PBS and 0.4 mL of 0.5% Trypan blue solution. The samples were mixed thoroughly, incubated at 23 °C for 20 min, and then 400 cells were counted by a light microscope (Olympus, Tokyo, Japan) for calculating the cell survival. Each experiment was repeated three times.

### 2.3. Western Blotting

Cells were harvested and washed with PBS, lysed on ice for 30 min using commercial protein extraction solution (TAKARA, Tokyo, Japan), and then centrifuged at 12,000× *g* for 10 min at 4 °C. The supernatants were collected, and the protein concentrations were measured using the commercial protein assay kit (Bio-Rad Laboratories, Inc., Hercules, CA, USA). Proteins were separated by sodium dodecyl sulfate–polyacrylamide gel electrophoresis (SDS-PAGE) and transferred to Immobilon P membranes (Millipore, Billerica, MA, USA). Membranes were blocked in 4% non-fat milk, then incubated with primary antibodies overnight at 4 °C. The catalog numbers and dilutions of all primary antibodies are as follows. Antibodies for caspase-3 (ab13847), p53 (ab131442), PARP-1 (ab137653), phospho-H2A.X (ab 54722), caspase-8 (ab 25901), H2A.X (ab140498), and caspase-9 (ab2324) were obtained from Abcam (Cambridge, MA, USA). The antibodies were used at dilutions 1:500, 1:200, 1:2000, 1:100, 1:100, 1:200 respectively. The primary antibodies for actin (61R-1159) (dilutions 1:200) was purchased from Fitzgerald Industries International, Inc. (Acton, MA, USA), Bax (2772) and PUMA (12450) were purchased from Cell Signaling Technology (Danvers, MA, USA) that were used at dilutions 1:1000 and 1:200. Then proteins were incubated with horseradish peroxidase-conjugated secondary antibodies for 2 h at 23 °C.

The protein bands were detected using the ECL Western Blotting Analysis System (Bio-Rad, Philadelphia, PA, USA). Chemiluminescent signals were examined by ImageQuant LAS 4000 (Bio-Rad, Philadelphia, PA, USA). Each experiment was repeated three times.

### 2.4. Apoptosis Assessment by DAPI Staining and TUNEL Assay

HCC cells were cultured on the glass slides for 12 h and treated with acetylshikonin (ASH) for 24 h at different concentrations. The HCC cells were cultured for 1, 2 and 3 days in a humidified atmosphere of 4% CO_2_ at 36 °C. Cells were fixed in a 4% formaldehyde solution in PBS and then permeabilized with Triton X-100 (0.1% in PBS) after incubation. Then, cells were stained with 4′, 6-diamidino-2-phenylindole (DAPI) in PBS (2.5 μg/mL) and allowed to stand for 20 min away from light. Finally, morphological changes were analyzed by fluorescence microscopy (Olympus, Tokyo, Japan). The apoptotic cells were also analyzed by using the In Situ Nick End-Labeling (TUNEL) assay using the ApopTag kit (Millipore, Billerica, MA, USA) principally following the supplier’s instruction. Images were captured using a Leica scanning confocal microscope (TCS SP5, Leica Microsystems, Ernst-Leitz-Strasse, Wetzlar, Germany).

### 2.5. ROS Production Assessment

For intracellular ROS visualization and determination, cells were incubated with 20 μM carboxy-H2DCFDA (Sigma-Aldrich, St. Louis, MO, USA) in RPMI for 40 min at 37 °C and washed with PBS twice. Fluorescence was visualized by using a fluorescent microscope (Olympus, Tokyo, Japan). The relative fluorescence intensity was detected by a microplate reader (SpectraMax; Molecular Devices, San Jose, CA, USA) with an excitation wavelength at 480 nm and an emission wavelength at 510 nm.

### 2.6. DNA Comet Assay

HepG2 cells with ASH vehicle were suspended in 1.5% agarose at 35 °C and layered on a frosted slide from the Trevigen Comet assay kit (Gaithersburg, MD, USA). The slides were submerged in pre-cooled lysis buffer containing 2.5 M NaCl, 100 mM ethylenediaminetetraacetic acid (EDTA), 1.5% Triton X-100, 15 mM Tris-HCl and 9% DMSO) and stored at 4 °C for 12 h. After washing the slides twice with enzyme buffer and then incubating them in enzyme buffer at 36 °C for 30 min, the slides were washed with enzyme buffer and denatured in cold NaOH (300 mM) with 1 mM EDTA in a horizontal electrophoresis chamber for 25 min. Electrophoresis voltage and currents were set as 20 V and 300 mA for 45 min. Then, slides were incubated in cold neutralizing buffer for 20 min and immersed in 75% ethanol for 3 min and then allowed to air dry. Finally, samples were stained with Vista Green DNA dye at 23 °C for 20 min away from light. The results were visualized by a fluorescent microscope (Olympus, Tokyo, Japan) and quantified by the Comet Assay software (Casplab, Gaithersburg, MD, USA). Tail moment was analyzed by calculating the percentage of tail DNA multiplied by the tail length.

### 2.7. siRNA Transfection

HepG2 cells were seeded at a density of 1 × 10^5^ cells/35-mm dish or 5 × 10^5^ cells/90-mm dish, and then the cells were transfected by Opti-MEM, containing 5 μL/mL Lipofectamine 2000 and 50 nM p53 or PUMA small (or short) interfering RNA (siRNA) for 10 h, as previously described [20]. The sequences of the siRNA are indicated in Table 1. HepG2 cells were collected 48 h after transfection. The efficiency of siRNA transfection was confirmed by western blot assay.

### 2.8. Orthotopic Transplantation Tumor Model of HCC Preparation and Treatment

HepG2 cells (2 × 10^6^) were subcutaneously injected into the flanks of 4-weeks-old male BALB/C nude mice. Once it reached a diameter of 1 cm, the subcutaneous tumor was cut into approximately 1 mm^3^ pieces and implanted into the capsule of left liver lobes at an angle of 20°. For surgical orthotopic liver tumor implantation, nude mice were anesthetized with an intravenous injection of 0.5% sodium pentobarbital (Nembutal, 25 mg/kg). Absorbable sutures were performed for skin closure. All of the animal protocols were approved by the Ethics committee for animal experiments in Kansas University (Approval number: AM (KU) 2018-0124), and the method was carried out following the approved guideline. To relieve pain after surgery, nude mice were received meloxicam (2 mg/kg) orally for seven days. Then the mice were randomized into two groups (n = 5). One group received ASH (1 µg/g body weight) and TRAIL (100 ng/g body weight) every two days via subcutaneous injection for four weeks. The control group mice received the same volume of vehicle (PBS + 0.01% BSA + 0.1% DMSO). The dosage of ASH and TRAIL were calculated based on previous research [7,21,22]. The tumor-bearing mice were sacrificed after four weeks treatment, and livers were excised and photographed. The numbers of tumor nodules in the livers of mice in different groups were analyzed by two independent researchers. The expressions of P53, PUMA and Bax in tumor tissue were analyzed by immunohistochemical assay.

### 2.9. Immunohistochemistry

Liver tumor sections were embedded in paraffin before being fixed in 8% buffered formalin solution for 12 h. Then the paraffin-embedded hepatic tumor tissues were analyzed for any expression of Bax, PUMA and p53 by immunohistochemistry as previously described [23]. Tumor tissue sections were incubated with primary anti-PUMA, anti-Bax from Cell Signaling Technology (Boston, MA, USA) and anti-P53 antibodies from Abcam (Boston, MA, USA). Incubation with an appropriate secondary antibody was followed by direct diaminobenzidine staining and light counterstaining with hematoxylin.

### 2.10. Kidney and Liver Function Tests

Blood samples were collected from the control and treated mice for analysis of liver and kidney functions at the end of the experiment following mice sacrificing. The blood urea nitrogen, serum creatinine, alanine transaminase and aspartate transaminase levels were determined by using a fully automated random access clinical chemistry analyzer (Beckman Synchron CX5, Foster, CA, USA).

### 2.11. Statistical Analyses

The data from above experiments are presented as the mean ± standard error of measurement (SE). Differences between groups were analyzed by one-way analysis of variance (ANOVA) and the Dunnett test for multiple comparisons (SigmaPlot for Windows version 12.0; Systat Software, Inc., San Jose, CA, USA). *p* values less than 0.05 were considered to represent a statistically significant difference.

## 3. Results

### 3.1. TRAIL Resistance in Human HepG2 Cell

To examine TRAIL sensitivity in HCC cells, HepG2 and Huh7 cells were exposed to TRAIL (0–200 ng/mL) for 8 h. The cell survival result indicated that TRAIL (50–200 ng/mL) significantly inhibited the cell viability of Huh7 cells dose-dependently (Figure 1A). The cell viability of Huh7 decreased by 34.35 ± 1.5%, 49.2 ± 2.97% and 60.32 ± 4.74% following 50, 100 and 200 ng/mL TRAIL treatments for 8 h, respectively. But the viability of HepG2 cells was approximately 91% after exposure to 200 ng/mL TRAIL. Furthermore, poly (ADP-ribose) polymerase-1 (PARP-1) cleavage, which is a validated indicator of cellular apoptosis, was only observed in Huh7 cells (Figure 1B). The apoptotic effects of TRAIL were further demonstrated by DAPI staining and the TUNEL assay.

HepG2 and Huh7 cells were subjected to DAPI staining after 100 ng/mL TRAIL treatment. Apoptotic cell death was compared between different cell lines. As shown in Figure 1C, in the DAPI staining image, distinct subcellular morphological changes of apoptosis (chromosome condensation) were observed in Huh7 cells, but not in HepG2 cells after the TRAIL treatment. For the TUNEL assay, the morphologic changes in apoptotic Huh7 cells were detected by a laser scanning confocal microscope after TRAIL treatment (Magnification× 200), which indicated DNA fragmentation within the Huh7 cells, while no fluorescence signal has been detected in the HepG2 group. These results indicated that Huh7 cells were sensitive to apoptosis-induced by TRAIL treatment, while HepG2 cells were resistant to TRAIL, which is consistent with the previous studies [24].

### 3.2. The Synergetic Effects of ASH and TRAIL on HCC Cells Apoptosis

We next determined whether applying ASH could induce cell death in a HepG2 cell. HepG2 cells were treated with ASH (0–10 μM) for 8 h, and cell survival rates were examined by the Trypan blue dye exclusion assay. Our data showed that 2.5 μM ASH used alone could not reduce the cell viability of this HepG2 cell (Figure 2A). Interestingly, 2.5 μM ASH combination with a low dose of TRAIL (50 ng/mL) could significantly suppress cells’ viability of HepG2 cells (Figure 2B). Figure 2C confirms that no obvious cleavages of PARP-1 were detected after ASH (1–5 μM) or TRAIL (50 ng/mL) exposure, respectively. In contrast, non-cytotoxic doses of ASH (2.5 μM) combined with 50 ng/mL TRAIL significantly promoted the cleavage of PARP-1 in HepG2 cells. To our surprise, ASH combined with TRAIL did not influence the cleavage of PARP-1 in a normal human hepatocyte LO2 cell (Figure 2D). In addition, DAPI staining and TUNEL assay clearly indicated the induction of apoptotic cell death in HepG2 cells after being co-treated with 50 ng/mL TRAIL and 2.5 μM ASH (Figure 2E).

### 3.3. Combination Therapy with TRAIL and ASH Activates Caspases Signaling Pathway

Next, the underlying mechanisms as to how TRAIL-mediated apoptosis was enhanced in HepG2 cells by ASH were investigated. We examined the cleavage of PARP-1, caspase-9, caspase-3 and caspase-8 in HepG2 cells to explore the regulation of the apoptotic signaling pathway after TRAIL and ASH treatment. No obvious cleavage of Caspase-3/-8/-9 or PARP-1 were detected following treatment with 2.5 μM ASH or 50 ng/mL TRAIL, respectively in this HepG2 cell (Figure 3A). In contrast, TRAIL (50 ng/mL) and ASH (2.5 μM) combination therapy lead to significant caspases and PARP-1 cleavages time-dependently (Figure 3A). In addition, the cleavages of caspases were increased by ASH dose-dependently (Figure 3B). Several caspases inhibitors such as zlETD-fmk, zlEHD-fmk and zDEVD-fmk were applied to validate the potential role of caspases cleavages in HepG2 cell survival after combination treatment.

Our data demonstrated that both the cleavage of PARP-1 and apoptosis in HepG2 cells were reversed by caspases inhibition (Figure 3C). In general, activation of caspases signaling might have contributed to apoptosis in the HepG2 cell mediated by non-cytotoxic doses of TRAIL and ASH.

### 3.4. ASH Promotes ROS Production in HepG2 Cells

It is widely accepted that the reactive oxygen species (ROS) plays a pivotal role in cell apoptosis. Thus, we assessed the effects of ASH and TRAIL on the intracellular redox status of HepG2 cells after 48 h treatment. Firstly, we detected the cellular ROS production after ASH treatment via applying the CARBOXY-H_2_DCFDA fluorescence probes. Figure 4A indicates that HepG2 cells pretreated with H_2_O_2_ (positive control) or ASH (1, 2.5 μM) exhibited an obvious fluorescence signal compared to control groups observed under a fluorescence microscope. The relative fluorescence intensity was enhanced by ASH according to the results from the fluorescence plate reader, which indicated that ASH may promote ROS production dose-dependently (Figure 4B). The maximum value of relative fluorescence intensity was presented at 20 min after ASH (2.5, 5 μM) treatment. Then, the relative fluorescence intensity quickly decreased and achieved a minimal value after ASH treatment 60 min later. However, the fluorescence intensity climbed again after ASH treatment for four hours (Figure 4C). The above data indicated that ASH increased the cellular ROS level in a biphasic pattern in the HepG2 cell.

To explore the potential role of ROS in ASH- and TRAIL-induced HepG2 cell apoptosis, cells were exposed to NAC (ROS inhibitor), and then these cells were treated with TRAIL (50 ng/mL) and ASH (2.5 μM). Figure 4D shows that 50 ng/mL TRAIL did not have any effect on ROS production based on the changes of fluorescence intensity. In addition, 4 mM NAC might decrease the ROS level induced by 2.5 μM ASH (Figure 4D), and reverse cell death caused by ASH and TRAIL combination treatment in a human HepG2 cell (Figure 4E). ROS can modify the cysteine residues of p53, a tumor suppressor, leading to conformational changes that affect its transcriptional activity [25]. ASH-induced apoptotic cell death has been associated with the up-regulating of p53 and PUMA expression in an HCC cell [16]. Thus, to reveal the mechanisms of ROS-mediated apoptosis by combination treatment with ASH and TRAIL, the Western blotting assay was applied to examine the cleavage of PARP-1 and the expression of p53 and PUMA in HepG2 cells. As shown in Figure 4F, TRAIL (50 ng/mL) and ASH (2.5 μM) synergistically increased the cleavage of PARP-1 and up-regulated the expression of p53 and PUMA in the HepG2 cell. However, 4 mM NAC alleviated the effects of ASH + TRAIL on the cleavage of PARP-1 and reversed the increasing of p53 and PUMA expression. In conclusion, ASH and TRAIL combination treatment may trigger the ROS-mediated intrinsic apoptosis pathway via increasing the expression of p53 and PUMA in the HepG2 cell.

### 3.5. ASH Caused DNA Damage in HepG2 Cells

ROS may lead to mutations of genes and chromosomes by DNA double strand breaks in the cell, which may further induce cell apoptotic death. To evaluate the DNA damage induced by ASH treatment, a comet assay (single-cell gel electrophoresis) was applied to measure DNA strand breaks in HepG2 cells. Figure 5A shows significant difference in tail length (length of DNA migration) after 2.5 µM ASH exposure 20 min later, which suggested that ASH could induce DNA damage in HepG2 cells. Above results indicated that ASH could induce DNA double strand breaks in HepG2 cells and trigger subsequent apoptotic cell death. When a double-strand break occurs in DNA, a sequence of events occurs in which the H2A histone family member X (H2AX) becomes phosphorylated on serine 139 [23,26]. Thus, we detected the expression of phospho-H2A.X-Ser139 and H2A.X to further confirm ASH induced DNA damage. Figure 5B,C showed that ASH time- and dose-dependently facilitated H2A.X phosphorylation on Ser-139 in HepG2 cell. In addition, the expression of TRAIL receptors (DR-4 and DR-5) in TRAIL-resistant HepG2 cells were unaltered after treatment with 2.5–10 µM ASH (Figure 5D). These results indicated that ASH might promote ROS production and DNA double-strand breaks, as well as the H2A.X phosphorylation on Ser-139, which might further activate P53 and trigger apoptosis in cancer.

### 3.6. Involvement of p53 and PUMA in ASH-Induced TRAIL Sensitization

It has been recognized that p53 phosphorylation could affect the stabilization of itself [27]. Interestingly, our results showed that 2.5 µM ASH can induce p53phosphorylation at Ser15, Ser392 and Ser46 residues, which facilitated the stabilization and accumulation of p53 in HepG2 cells (Figure 6A). The P53 up-regulated modulator of apoptosis (PUMA) is a downstream target of p53. Previously, study has shown that p53 activation can up-regulate PUMA and induce cell apoptosis after ASH treatment [16]. Herein, we further explored the potential role of PUMA and p53 in ASH- and TRAIL-mediated apoptotic cell death.

Figure 6B further confirms that ASH significantly increased the expressions of p53 and PUMA in a dose-dependent manner. A significant increase of PUMA and p53 expression is observed by the synergistic therapy of TRAIL (50 ng/mL) and a non-cytotoxic dose of ASH (Figure 6C). For further confirming the critical role of p53 and PUMA in ASH-induced TRAIL sensitization, RNA interference (RNAi) was applied to knock down the expression of p53 and PUMA. Figure 6D shows that at the 48-h time point after PUMA or p53 siRNA transfection, ASH-mediated TRAIL sensitization was reversed in PUMA- or p53 siRNA-transfected cells, as indicated by the alleviated PARP-1 cleavage. The DAPI staining results were consistent with the Western blotting experiments (Figure 6E). In general, the above results demonstrated that p53 and PUMA might play critical role in ASH-induced TRAIL sensitization and apoptosis. To further confirm the involvement of p53 in TRAIL- and ASH-induced apoptosis of different HCC cell lines, Hep3B, another TRAIL-resistant HCC cells, were performed in our study. Two Hep3B HCC cell lines, including p53+/+ and p53−/−, were exposed to TRAIL and ASH treatment. Our results indicated that ASH can synergize with TRAIL and induce cytotoxicity as well as up-regulate PARP-1 cleavage in Hep3B p53+/+ cells instead of Hep3B p53−/− cells (Figure 7A,B). In another experiment, two Hep3B cell lines (Hep3B PUMA+/+) and (Hep3B PUMA−/−) were applied to further evaluate the potential role of PUMA in ASH- and TRAIL-induced HCC apoptosis. Figure 7C,D demonstrate that ASH may sensitize TRAIL-induced apoptotic cell death and promote the cleavage of PARP-1 in the Hep3B PUMA+/+ cell instead of the Hep3B PUMA−/− cell. In summary, these results revealed that increased expression of PUMA or p53 contributed to sensitize HCC cells to TRAIL-induced apoptosis by ASH.

### 3.7. Bax Contributed to ASH and TRAIL Induced Apoptosis

After PUMA activation, it will further interact with anti-apoptotic Bcl-2 family members, thus freeing Bax which is then able to signal apoptotic cell death to the mitochondria [19]. To verify whether Bax contributed to ASH- and TRAIL-induced apoptosis, HepG2 Bax+/− and HepG2 Bax−/− cells were used in our study. As shown in Figure 8A,B, TRAIL-induced cytotoxicity and PARP-1 cleavage were facilitated by 2.5 μM ASH synergistic treatment in the HepG2 Bax+/− cell, but not in the HepG2 Bax−/− cell. Interestingly, the synergistic treatment remarkably increased the upstream activators of Bax, such as p53 and PUMA in both cell lines (Figure 8B). In addition, the DAPI staining assay also clearly indicated the induction of apoptotic cell death in HepG2 Bax+/− cells after combination treatment with TRAIL (50 ng/mL) and 2.5 μM ASH (Figure 8C).

### 3.8. ASH and TRAIL Inhibits Tumor Growth in Orthotopically Transplanted Mouse HCC

We next sought to determine whether ASH and TRAIL combination treatment can inhibit tumor growth in orthotopically transplanted mouse HCC. Tumor-bearing mice treated with ASH (1 µg/g body weight) + TRAIL (100 ng/g body weight) every two days via subcutaneous injection for four weeks, showed 2.7-fold reduction in the tumor nodules number in livers compared to our control group (*p* < 0.05 Figure 9A). For detecting the potential side effect of ASH + TRAIL, we examined the body weight of mice during the treatment. As shown in Figure 9B, there were no obvious changes in body weight between the two groups (*p* < 0.05). We further detected the effects of ASH + TRAIL on kidney and liver functions. We did not find significant differences on blood urea nitrogen, serum creatinine, alanine transaminase and aspartate transaminase levels between the two groups (*p* < 0.05) (Table 2). Together, these results suggest that ASH + TRAIL has no significant side effects in mice. In addition, the IHC results showed that the number of positive cells and the intensity of staining for p53, Bax and PUMA were significant higher in liver cancer tissue in the ASH + TRAIL group compared with vehicle treated controls. (*p* < 0.05 Figure 9C).

## 4. Discussion

Apoptosis can be triggered by extracellular stimuli (extrinsic pathway) or irritation within the cells (intrinsic pathways). For intrinsic apoptosis, the cell death was induced by cell stress such as DNA damage and subsequently p53 activation. For extrinsic apoptosis the cell kills itself due to signals from other cells mediated by binding to death ligands and their receptors. Caspases orchestrate both extrinsic and intrinsic apoptosis by activating target protein cleavage [28]. TRAIL, also recognized as Apo2L, belongs to the TNF superfamily, which could induce cell apoptosis via activating the extrinsic apoptosis pathway. The pre-treatment of the cancer cell by small molecules inhibitor has been shown to improve the sensitivity of TRAIL-induced apoptosis while sparing the normal cell [29]. These novel agents include the mammalian target of the rapamycin (mTOR) inhibitor [30], BCL-2 inhibitor [31], histone deacetylases (HDAC) inhibitor [32] and proteasome inhibitor [33], which have been used for combination with TRAIL to suppress the specific signal molecule that might synergistically promote a TRAIL-induced extrinsic apoptosis pathway. In this study, we found that non-cytotoxic dosage of ASH might sensitize HepG2 cells to TRAIL-induced apoptosis via up-regulating the expression of p53, PUMA and Bax through oxidative DNA damage induced by ROS. Mitochondria-mediated activation of caspase-9 was involved in the intrinsic apoptosis signal pathway induced by ASH via the promotion of ROS production, while death-receptor mediated activation of caspase-8 might contribute to the extrinsic apoptosis signal pathway by TRAIL (Figure 10).

TRAIL therapy has been introduced for cancer treatment by inducing an extrinsic apoptosis pathway for more than twenty years. However, various tumor cells showed resistance to TRAIL treatment [6]. Herein, our data showed that the liver cancer cells Huh7 were sensitive to TRAIL-induced apoptosis, while HepG2 cells were resistant. Above results were consistent with previous research on TRAIL-sensitive or -resistant HCC cells [31].

More importantly, our data indicated that non-toxic dosage of ASH in combination with TRAIL significantly induced apoptotic cell death in the HepG2 cell. These findings suggested that ASH might have synergistic or sensitizing effects on TRAIL-mediated apoptosis. In the intrinsic pathway of apoptosis, opening the permeability transition pore complex on the mitochondrial membrane plays a critical role in the subsequent release of cytochrome C, formation of apoptosome and in activating caspase. Caspases are a family of cysteine aspartyl proteases which constitutes the effector arm of the apoptotic machinery. When caspases are activated, they will trigger the cleavage of various intracellular proteins to bring programed cell death by apoptosis [34]. Our data suggested that ASH and TRAIL synergistically up-regulated caspase-3, -8 and -9 expressions, which confirmed the pivotal role of caspases in the apoptosis of HCC cells. ROS can open the pore via pore-destabilizing proteins’ activation such as Bax [11]. In our study, an increased intracellular ROS level was observed after ASH exposure. In addition, ASH significantly induced DNA double strand breaks in our HepG2 cell. Combination therapy with non-toxic doses of TRAIL and ASH resulted in the activation of caspase and the cleavage of PARP-1 in HepG2 cells, which may contribute to the ROS-induced intrinsic pathway of apoptosis. Interestingly, the application of an antioxidant such as NAC obviously suppressed the intracellular ROS level and the cleavage of PARP-1, thus alleviating the cancer cells’ apoptosis induced by the synergistic treatment with ASH and TRAIL. Furthermore, NAC also blocked the expression of p53 and PUMA in the HepG2 cell, which would inhibit cell apoptosis. PUMA is an important mediator of p53-dependent apoptosis, which can transduce death signals to the mitochondria, where it indirectly activates Bax and subsequently induces mitochondrial dysfunction and caspase activation [28,35]. Here we showed an increased expression of Bax and PUMA in HCC cells following exposure to ASH and TRAIL. P53 and PUMA silencing or Bax gene deficiency could reverse ASH-induced TRAIL sensitization in HCC. Above data suggested that ROS played a critical role in DNA damage and activating p53/PUMA/Bax signaling, thus leading to the permeabilization of the mitochondrial outer membrane and the activation of caspases as well as sensitization of HCC cells to TRAIL-induced apoptosis by ASH. Although several natural compounds or small molecules have been reported to induce cell death by promoting ROS production, their mechanisms as to how ROS is induced are still largely unclear. Therefore, the mechanisms underlying the pharmacological activity of ASH in increasing the intracellular ROS level will be further studied in our future research.

Next were further examined the protective effects of ASH and TRAIL in the orthotopically HCC-implanted mice. The in vivo results indicated that the combination therapy may inhibit HCC development without significant cytotoxicity to mice. The immunohistochemistry (IHC) analysis for p53, PUMA and Bax expression from tumor tissue also confirmed our in vitro results. In summary, we demonstrated that HCC cells co-treated with ASH and TRAIL will result in ROS production, DNA double strand breaks and p53-mediated PUMA and Bax up-regulation, followed by caspases activation and consequently inducing apoptosis in the HepG2 cell while sparing the normal hepatic LO2 cell. Despite our encouraging findings in this study, several questions remain, such as how ROS is induced by ASH, and the safety and efficacy of our combination treatment of ASH and TRAIL on cancer patients. In addition, whether this combination has a “synergistic” effect on the inhibition of HCC cells’ survival should be further studied by in silico-based automated simulation of synergism, at all dose or effect levels, as previously described [36]. These questions need to be carefully answered by our future studies.

## Figures and Tables

**Figure 1:** The tumor necrosis factor-related apoptosis-inducing ligand (TRAIL) inhibits cell viability and induces apoptosis in Huh7 cells. (**A**) The HepG2 and Huh7 cells’ survival rates were detected by the Trypan blue dye exclusion assay following TRAIL treatment (0–200 ng/mL) for 8 h. Our control group received an equal amount of vehicle (PBS + 0.01% BSA) * *p* < 0.05; ** *p* < 0.01. (**B**) After TRAIL treatment (0–200 ng/mL), western blot was applied to examine PRAP-1 cleavage in HepG2 and Huh7 cells. (**C**) HepG2 and Huh7 cells were subjected to 4′,6-diamidino-2-phenylindole (DAPI) staining. Apoptotic cell death was compared between different cell lines after 100 ng/mL TRAIL treatments. Chromatin condensation of the tumor cells was shown with white arrows observed by fluorescence microscopy. For the terminal deoxynucleotidyl transferase dUTP nick end labeling (TUNEL) assay, the morphologic changes in apoptotic hepatocellular carcinoma (HCC) cells (green) were detected by a laser scanning confocal microscope (Magnification× 200).

**Figure 2:** Non-apoptosis-inducing doses of acetylshikonin (ASH) reversed the resistance to TRAIL-induced apoptosis in the HepG2 cell. (**A**) After ASH treatment (1–10μM) or vehicle (0.1% dimethyl sulfoxide (DMSO)) for 8 h, cell survival rates were examined in HepG2 cells. (**B**) HepG2 cells were treated with ASH (0–10μM) and TRAIL (50 ng/mL), and survival rates were detected by the Trypan blue dye exclusion assay. * *p* < 0.05; ** *p* < 0.01 (**C**) Human hepatoma HepG2 cells and (**D**) normal hepatocytes LO2 cells were exposed to TRAIL (50 ng/mL) and 2.5 μM ASH for 12 h. Cell lysates were prepared after treatment and analyzed by Western blotting assay using antibodies specific to PARP-1and Actin. (**E**) Cell apoptosis was assessed by our TUNEL assay and DAPI staining (Magnification× 200).

**Figure 3:** Combination therapy with ASH and TRAIL results in the activation of caspase in the HepG2 cell. (**A**) The cleavage of caspases and PARP-1 in HepG2 cells were analyzed via Western blotting after following 4–24 h treatment with 2.5 µM ASH and/or 50 ng/mL TRAIL, and the control group received an equal amount of vehicle (PBS + 0.01% BSA + 0.1% DMSO). (**B**) Western blotting was applied to determine the cleavage of caspase family members in HepG2 cells after treatment with 0.5–2.5 µM of ASH and 50 ng/mL TRAIL for 12 h. (**C**) The specific caspases inhibitors were applied to HepG2 cells to block the caspase pathway. Then the cells were exposed to 2.5 µM ASH and/or TRAIL 50 ng/mL for 12 h. Cells’ survivals were assessed via the Trypan blue dye exclusion assay and Western blotting was applied to determine the cleavage of PARP-1. ** *p* < 0.01.

**Figure 4:** ASH-induced ROS production in a HepG2 cell. (**A**) ROS production in HepG2 cells was analyzed by fluorescence microscopy. Cells were treated with H2O2 (positive control) or ASH (1, 2.5 μM) for 60 min and labeled with CMH2DCFDA (20 μM/L) for 20 min. The positive control group or ASH (2.5, 5 μM) group showed significant higher fluorescence intensity as compared to the vehicle (PBS + 0.01% BSA) control group. (**B**) After exposure with ASH (2.5, 5 μM) for various times, the intracellular ROS production in HepG2 cells was analyzed by the relative fluorescence intensity. * *p* < 0.05; ** *p* < 0.01; *** *p* < 0.001 (**C**) HepG2 cells were labeled with CMH2DCFDA after treating with ASH (2.5, 5 μM) for different times. ROS productions at different time-points were quantified by the relative fluorescence intensity using the fluorescence plate reader. * *p* < 0.05 (**D**) Pretreated with N-acetyl-l-cysteine (NAC) (ROS inhibitor) significantly decreased the ROS level induced by ASH (25 μM), and (**E**) reversed ASH- and TRAIL-mediated HepG2 cell death. * obvious changes between ASH and TRAIL + ASH group (*p* < 0.05). ** Obvious changes between NAC+ TRAIL + ASH group and TRAIL + ASH group (*p* < 0.01). Control group received an equal amount of vehicle (PBS + 0.01% BSA + 0.1% DMSO). (**F**) Western blotting was applied to determine the cleavage of PARP-1 and the expression of p53, and the p53 upregulated modulator of apoptosis (PUMA) after pretreatment of NAC in combination with ASH and/or TRAIL.

**Figure 5:** ASH promotes DNA damage and H2A.X phosphorylation in HepG2 cell. (**A**) DNA Damage caused by 1–2.5 µM ASH was measured by the Comet Assay for 20 min. Tail moment was used to measure the double strand breaks by calculating the percentage of tail DNA x tail length. * *p* < 0.05; ** *p* < 0.01. (**B**) HepG2 cells were pretreated with 1–10 µM ASH for 12 h, the expression of phospho-H2A.X-Ser^139^ and H2A.X were analyzed by Western blot assay. Control group received an equal amount of vehicle (0.01% DMSO). (**C**) HepG2 cells were pretreated with 2.5 µM ASH for 0, 1, 2, 4, 8, 16, and 24 h. The expressions of phospho-H2A.X-Ser139 and H2A.X were analyzed by Western blot assay. (**D**) HepG2 cells were pre-incubated with ASH at various dosages for 12 h. The expression of DR-4 and DR-5 was evaluated by Western blotting assay.

**Figure 6:** ASH promotes phosphorylation and accumulation of p53 and increases PUMA expression. (**A**) HepG2 cells were exposed to 2.5 µM ASH for 1, 2, 4, 8, 16 and 24 h, phosphorylation of p53 at Ser46, Ser392 and Ser15 residues were analyzed by Western blotting assay). Control group received an equal amount of vehicle (0.1% DMSO). (**B**) HepG2 cells were exposed to 1, 2.5, 5, 10 µM ASH for 12 h, the expression of PUMA and p53 protein were analyzed by western blotting assay. (**C**) HepG2 cells were exposed to 1, 2.5, 5 µM ASH with or without 50 ng/mL TRAIL for 12 h, PUMA and p53 protein expression were analyzed by western blotting assay. (**D**) Small interfering RNA (siRNA) has been used to specifically silence PUMA or p53; 48 h after transfection, the HepG2 cells were exposed to 5 µM ASH with or without 50 ng/mL TRAIL for 12 h. The cleavage of PARP-1 and the expression of p53 and PUMA were analyzed via Western blotting assay. (**E**) DAPI staining test was performed to assess the apoptosis-inducing effects of ASH and TRAIL combination therapy in HepG2 cells after P53 or PUMA siRNA transfection. Chromatin condensation of the tumor cells was shown with white arrows observed by fluorescence microscopy (Magnification× 200).

**Figure 7:** ASH reverses TRAIL resistance and induces apoptosis in Hep3B cells by targeting p53 and PUMA. (**A**,**B**) Wild-type and p53−/−Hep3B cells or (**C**,**D**) wild type and PUMA−/−Hep3B cells were pretreated with ASH (2.5 μM) and TRAIL (50 ng/mL) for 12 h. Control group received an equal amount of vehicle (PBS + 0.01% BSA + 0.1% DMSO). Cell survivals were detected by the Trypan blue dye exclusion assay. The cleavage of PARP-1 and the expression of p53 or PUMA were analyzed via Western blotting. * *p* < 0.05.

**Figure 8:** Bax contributed to apoptosis induced by ASH and TRAIL. (**A**,**B**) 2.5 µM ASH and 50 ng/mL TRAIL were exposed to HepG2 Bax+/− and HepG2 Bax−/− for 8 h. Control group received an equal amount of vehicle (PBS + 0.01% BSA+0.1% DMSO). Cells’ survivals were detected by the Trypan blue dye exclusion assay. The cleavage of PARP-1 and the expression of PUMA, p53 and Bax were analyzed by the Western blotting assay * *p* < 0.05. (**C**) The DAPI staining test was performed to assess apoptosis-inducing effects of ASH and TRAIL combination therapy in HepG2 Bax+/− and HepG2 Bax−/− cells. Chromatin condensation of the tumor cells was shown with white arrows observed by fluorescence microscopy (Magnification× 200).

**Figure 9:** ASH and TRAIL combination treatment inhibits tumor growth in orthotopically transplanted mouse HCC (**A**) The amount of tumor nodules in livers from tumor-bearing mice after ASH (1 µg/g body weight) and TRAIL (100 ng/g body weight) combination treatment via subcutaneous injection for four weeks. Mice in the control group received an equal amount of vehicle (PBS + 0.01% BSA + 0.1% DMSO) (** *p* < 0.01). (**B**) Body weight of tumor-bearing mice was examined during treatment. No obvious loss in body weight could be detected, suggesting ASH (1 µg/g body weight) + TRAIL (100 ng/g body weight) might not have significant cytotoxicity in vivo. (**C**) P53, PUMA and Bax expression were assessed by immunostaining; the final immunostaining score was calculated by multiplying the intensity score with the percentages of positive cell observed by electron microscopy at 200× magnification. The intensity of staining was scored by three independent researchers as 0 = no staining, 1 = weak staining and 2 = significant staining. Cancer cells in four fields were selected randomly and scored based on the percentage of positive staining cell (** *p* < 0.01).

**Figure 10:** Diagram of molecular mechanisms underlying the synergic effects between ASH and TRAIL in promoting apoptotic cell death in HCC.

**Table 1:** Sequences for small (or short) interfering RNA (siRNA) transfection.

Gene Name	Gene Bank ID	siRNA Sequences
P53	AB082923	F: 5′-CUCCAUCUGGGAAUGACUU-3′ R: 5′-UAUCCAAUCUGAACUGGAC-3′
PUMA	AF354654	F: 5′-GUGCCAUUGCGAAUGAAUA-3′ R: 5′-ACUUCAUUCUCAAGUGACC-3′

**Table 2:** The effects of ASH+TRAIL on kidney and liver functions in mice.

Serum Chemistry	Control	ASH + TRAIL	*p*-Value
Blood urea nitrogen (mg/dL)	54.7 ± 4.97	49.8 ± 2.57	0.221
Serum creatinine (µmol/L)	105.48 ± 8.52	112.60 ± 7.58	0.647
Alanine transaminase (U/L)	59.78 ± 9.39	67.48 ± 12.81	0.569
Aspartate transaminase (U/L)	323.94 ± 71.4	380.15 ± 87.3	0.309
